# A Controlled Study of Continuous Lumbar Drainage of Fluid and Lumbar Puncture Drainage for Aneurysmal SAH after Intracranial Aneurysm Clipping

This article has been retracted.

**DOI:** 10.1155/2021/2827493

**Published:** 2021-08-20

**Authors:** Fei Duan, Guofei Wang, Xiaohu Ma, Yue Zhao, Xuanle Xu, Fada Dong

**Affiliations:** Department of Neurosurgery, The First People's Hospital of Xianyang, Xianyang, Shaanxi Province, China

## Abstract

**Objective:**

To analyze the different effects of Continuous Lumbar Drainage of fluid and lumbar puncture drainage for aneurysmal subarachnoid hemorrhage (SAH) after intracranial aneurysm clipping.

**Method:**

Seventy-five patients with aneurysmal SAH who underwent aneurysm clipping were retrospectively analyzed and were divided into two groups according to the different postoperative drainage methods. The lumbar spine group received lumbar puncture drainage, and the lumbar cistern group received lumbar pool continuous drainage to compare the efficacy.

**Result:**

The time to normalize intracranial pressure and headache relief after drainage treatment in the lumbar cistern group was shorter than that in the lumbar spine group. The GOS score was higher than that in the lumbar spine group, and the cerebral artery flow velocity and NIHSS score were significantly lower than those in the lumbar spine group (*P* < 0.05). The total effective rate of drainage treatment was 76.32% in the lumbar cistern group, which was higher than that in the lumbar spine group (54.05%) (*P* < 0.05). The total complication rate was 18.42% in the lumbar cistern group, which was lower than that in the lumbar spine group (40.54%) (*P* < 0.05).

**Conclusion:**

Continuous Lumbar Drainage of fluid after intracranial aneurysm clipping for aneurysmal SAH can control symptoms more rapidly, reduce neurological deficits, and improve prognosis than lumbar puncture. Also, the drainage is safer and more widely used.

## 1. Preface

Subarachnoid hemorrhage (SAH) is a type of craniocerebral diseases with a high incidence and severity, specifically a disease in which lesions in the superficial layers and base of the brain cause rupture of blood vessels and blood enters the subarachnoid space, eventually leading to abnormal intracranial pressure [1]. Statistics show that in all acute brain death diseases, the incidence of SAH is close to 10% [2]. It was found that diseases that may lead to cerebral hemorrhage may trigger SAH, and common causes include cerebrovascular malformations, intracranial aneurysms, anomalous vascular network disease at the base of the brain, and other related complications such as vasculitis and intracranial tumors [3].

Aneurysmal SAH is a common type of SAH. Acquired endosteal lesions of the arterial wall, congenital defects of the muscular layer of the arterial wall, and a combination of both are important factors in the development of aneurysms [4]. There are two main effects of incomplete intracranial aneurysm: one is born with abnormalities and the other is caused by living environment and lifestyle habits, and the latter is the main factor [5]. Intracranial aneurysm clipping is the main method of clinical treatment for diagnosed aneurysms, through which the blood supply to the aneurysm can be blocked to prevent rebleeding, in addition to keeping the aneurysm-carrying and blood-supplying arteries open and maintaining normal blood transport in brain tissue [6]. However, surgical treatment alone cannot completely remove the intracranial subarachnoid hemorrhage, and postoperative adjunctive drainage therapy must be performed to remove the clot.

Lumbar puncture has been widely used in the past, but it is more invasive, requires multiple punctures, and is not well accepted by patients. Continuous Lumbar Drainage of fluid (LCFD) is less invasive and has controlled drainage, which can prevent patients from needing to undergo repeated lumbar punctures and achieve long-lasting and continuous drainage of cerebrospinal fluid, while effectively controlling intracranial hypertension and facilitating targeted therapy at a later stage [7]. However, the application of LCFD may also lead to complications such as catheter occlusion, intracranial infection, nerve root irritation, intracranial hematoma, cerebrospinal fluid leakage at the puncture site, and intracranial pneumatosis [8]. Therefore, there is no uniform conclusion on which drainage method is more effective. In this study, a retrospective analysis of 75 patients with aneurysmal SAH was performed to compare the difference in the value of the application of these two drainage methods.

## 2. Information and Method

### 2.1. Information

The clinical data of 75 patients with aneurysmal SAH in our hospital were retrospectively analyzed. The study passed the ethical approval of the hospital where it was conducted. Inclusion criteria were as follows. (1) Patients who met the diagnostic criteria for aneurysmal SAH [9]. (2) Patients who were treated with intracranial aneurysm clipping. (3) Patients who had postoperative need for drainage. (4) Hunt–Hess classification [10] being grade III-IV. (5) Patients who were older than 18 years. (6) Patient's family or delegate having signed the study consent form. Exclusion criteria were as follows. (1) Patients who had contraindications to CT and MRI examinations. (2) Patients who had contraindications to surgery. (3) The expected survival time of patients after surgery not exceeding 12 months. (4) Patients who had severe liver dysfunction. (5) Hunt–Hess classification being grade IV-V. (6) The time between surgeries after onset exceeding 3 days.

### 2.2. Method

All patients were admitted to the ICU and were treated with fluid rehydration, water-electrolyte balance maintenance, blood pressure control, anti-vascular spasm by nimodipine, and cranial pressure control by mannitol. Various preoperative examinations were performed quickly, and intracranial aneurysm clipping was implemented within 3 days of admission. The operation was performed under general anesthesia, with a modified pterygoid approach. The head was fixed, the cerebral lobes were exposed, and the aneurysm was separated under the microscope. The aneurysm clip is selected according to the direction and size of the aneurysm, and if necessary, the aneurysm-bearing artery is blocked to ensure a satisfactory clip effect. During the operation, ultrasound is used to monitor the aneurysm clipping. If the aneurysm is combined with brain herniation, debridement and decompression should be performed after the aneurysm is clipped and the hematoma is removed. It was noted that the peripheral aneurysm hematoma was not removed temporarily before the aneurysm was clipped to prevent the aneurysm from rupturing. Anti-vascular spasm, hemodilution, and intracranial pressure elevation were given after the surgery. Patients in both groups received different methods of postoperative drainage.

In the lumbar spine group, conventional lumbar puncture was performed for drainage. A lumbar puncture was performed once every 2 days, and about 30 ml of cerebrospinal fluid was withdrawn each time. 4 punctures were performed continuously for drainage.

In the lumbar cistern group, LCFD was implemented by entering the needle in the L3-4 and L4-5 interspace of the lumbar spine. Complete the guidewire placement after puncturing the needle to the caudal subarachnoid space and place it into the subarachnoid space after skin expansion, pull out the guidewire when the depth of the puncture needle was maintained at 5–8 cm, clip the secondary tube after both the primary and secondary tubes flowed out the cerebrospinal fluid, make the connection of the main tube and drainage bag, adjust the drainage flow and flow rate, and control the daily drainage volume at 150–200 ml. The drainage should be continued for 8 days.

### 2.3. Observed Indicators

The time to normalization of intracranial pressure and the time to relief of headache between the two groups were compared.

The Glasgow Outcome Scale (GOS) [11] was used to evaluate the recovery of patients after drainage. 1 means death. 2 means vegetative survival status. 3 means severe disability. 4 means mild disability. 5 means good recovery.

The cerebral artery flow velocities before and after drainage treatment were compared between the two groups. If the cerebral artery flow velocity was between 120 cm/s and 140 cm/s, it indicated that patients had mild cerebral vasospasm. If the cerebral artery flow velocity was between 141 cm/s and 200 cm/s, it indicated that patients had moderate cerebral vasospasm. If the cerebral artery flow velocity was above 200 cm/s, it indicated that patients had severe cerebral vasospasm.

The neurological deficits before and after drainage treatment were compared between the two groups and evaluated using the Neurologic Impairment Score (NIHSS) [12] scale with 11 items, such as level of consciousness, gaze, visual field, facial palsy, upper limb movement, lower limb movement, limb ataxia, sensory, language, dysarthria, and neglect. Scores were 0–42, with higher scores indicating more severe neurological deficits.

The total effective rate of the two groups after drainage treatment was compared. Cured: all clinical symptoms disappeared after treatment, the neurological deficit score decreased by 90%, and the GOS classification was grade 5. Improved: the clinical symptoms decreased after treatment, the neurological deficit score decreased by 40%–89%, and the GOS classification was grade 4. Ineffective: the clinical symptoms did not change significantly or further aggravated after treatment, the neurological deficit score decreased by less than 40%, and the GOS grade was 1–3. Total effective rate is equal to cure rate plus improvement rate.

The incidence of complications during drainage between the two groups was compared.

### 2.4. Statistical Method

All data were analyzed using SPSS 23.0, and [*n* (%)] represents count data. In *X*^2^ test, ($\bar{x}$ ± *s*) represents measurement data. Independent sample *t* test is performed for comparison between groups, and paired *t* test is performed for comparison before and after within groups. ANVOA analysis is for multipoint comparisons. The data of *F*-test and graphs were processed by GraphPad Prism software (version 9.0). *P* < 0.05 was considered statistically significant.

## 3. Result

### 3.1. General Information

There was no statistical difference between the lumbar cistern group and the lumbar spine group for proportion by gender, Hunt–Hess grade, and aneurysm site (*P* > 0.05). There was no statistical difference between the lumbar cistern group and the lumbar spine group for mean age, time between surgeries, and longest diameter of aneurysm (Table 1 and Figure 1).

### 3.2. Time to Normalization of Intracranial Pressure and Relief of Headache

The time to normalization of intracranial pressure in the lumbar cistern group after receiving LCFD was (10.42 ± 2.94) days, which was shorter than that in the lumbar spine group that received lumbar puncture (14.75 ± 4.13) days. The time to headache relief in the lumbar cistern group was (11.19 ± 2.76) days, which was significantly shorter than that in the lumbar spine group ((15.71 ± 4.92) days), and all differences were statistically significant (*P* < 0.05) (Figure 2).

### 3.3. Prognostic GOS Evaluation Result

There was no statistically significant difference in the prognostic GOS score between the lumbar cistern group and the lumbar spine group before receiving drainage treatment (*P* > 0.05). The GOS scores were higher in both groups after receiving the corresponding drainage treatment than before the group treatment, and the difference was statistically significant (*P* < 0.05). The GOS scores were significantly higher in the lumbar cistern group after receiving drainage treatment than in the lumbar spine group, and the difference was statistically significant (*P* < 0.05) (Figure 3).

### 3.4. Changes in Cerebral Artery Flow Velocity

The difference in cerebral artery flow velocity between the lumbar cistern group and the lumbar spine group before receiving drainage treatment was not statistically significant (*P* > 0.05). The cerebral artery flow velocity was significantly lower in both groups after receiving the corresponding drainage treatment than before the group treatment (*P* < 0.05). The cerebral artery flow velocity was significantly lower in the lumbar cistern group after receiving drainage treatment than that in the lumbar spine group, and the difference was statistically significant (*P* < 0.05) (Figure 4).

### 3.5. Changes in Neurological Deficits

There was no statistically significant difference in NIHSS scores between the lumbar cistern group and the lumbar spine group before receiving drainage treatment (*P* > 0.05). The NIHSS scores were significantly lower in both groups after receiving the corresponding drainage treatment than before treatment in the group (*P* < 0.05). The NIHSS scores were significantly lower in the lumbar cistern group after receiving drainage treatment than those in the lumbar spine group, and the difference was statistically significant (*P* < 0.05) (Figure 5).

### 3.6. Total Efficiency of Drainage Treatment

Ten patients were cured, 19 improved, and 9 were invalid after receiving LCFD in the lumbar cistern group, with a total effective rate of 76.32%. 5 patients were cured, 15 improved, and 17 were invalid after receiving lumbar puncture in the lumbar spine group, with a total effective rate of 54.05%. The total effective rate of drainage treatment in the lumbar cistern group was significantly higher than that in the lumbar spine group, and the difference was statistically significant (*P* < 0.05) (Table 2).

### 3.7. Incidence of Complications

During the drainage treatment of 38 patients in the lumbar cistern group, 7 patients developed complications, including hydrocephalus (1), cerebral vasospasm (2), cerebral infarction (1), rebleeding (1), and other complications (2), with a total incidence of 18.42%. During the drainage treatment of 37 patients in the lumbar spine group, 15 patients developed complications, including hydrocephalus (2), cerebral vasospasm (4), cerebral infarction (3), rebleeding (2), and other complications (4), with a total incidence of 40.54%. The incidence of complications during drainage treatment in the lumbar cistern group was significantly lower than that in the lumbar spine group, and the difference was statistically significant (*P* < 0.05) (Table 3).

## 4. Discussion

Patients with low-grade aneurysmal SAH can be treated surgically with satisfactory results, but for patients with high-grade aneurysmal SAH, not only the cure rate of surgical treatment is not high but also the postoperative mortality rate is high. Currently, no specific treatment plan has been found for patients with high-grade aneurysmal SAH, and it is basically not suitable for conservative treatment due to the high rate of posttreatment complications. To summarize previous studies, it is important to not only treat patients with high-grade aneurysmal SAH aggressively but also control the residual blood accumulation to the greatest extent possible. Drainage is an effective method to reduce blood accumulation. It is very important to grasp the indications of drainage and choose the appropriate drainage method to ensure the drainage effect. The advantages of LCFD are that it can speed up the relief of meningeal irritation and shorten the time of cerebrospinal fluid clearing, reducing the pain caused by frequent lumbar puncture. Also, it can rapidly control the intracranial pressure of patients, reduce the risk of hydrocephalus and epilepsy, and ensure a higher success rate of puncture; thus, it can effectively control the outflow rate, reduce the trauma to patients and have higher patient acceptance [13, 14]. Reference [15] used LCFD in cerebrospinal fluid drainage and showed a reduction in intracanalicular cerebrospinal fluid pressure. Reference [14] used LCFD in the treatment of central nervous system disorders, which also showed good result.

In this paper, a controlled study was conducted to analyze the value of the two drainage modalities, and the result showed that when LCFD was performed after intracranial aneurysm clipping in the lumbar cistern group, patients had shorter time to normalize intracranial pressure and headache relief compared with the lumbar group that received lumbar drainage, in addition to higher GOS scores and lower cerebral artery flow velocity and NIHSS scores after treatment compared with the lumbar cistern group (*P* < 0.05). It indicates that LCFD used for aneurysmal SAH patients after intracranial aneurysm clipping can improve symptoms more rapidly, control neurological deficits, and improve prognosis. In this study, the total effective rate of drainage treatment in the lumbar cistern group was 76.32% and the total complication rate was 18.42%, which were better compared with the total effective rate of 54.05% and the total complication rate of 40.54% in the lumbar spine group (*P* < 0.05). This indicates that the LCFD method was chosen to obtain better treatment result compared with lumbar puncture drainage and to improve treatment safety. This is consistent with the result of similar studies [16–18]. Reference [19] also showed that patients in the lumbar cistern continuous drainage group recovered significantly better after treatment than the lumbar puncture group, and the disability and complication rate was significantly lower than that in the lumbar spine group (*P* < 0.05), which is consistent with the result of this study. Reference [20] confirmed that continuous drainage of the lumbar cistern group can achieve higher efficacy and safety compared with lumbar puncture group for the release of cerebrospinal fluid in the treatment of traumatic SAH.

The LCFD method applied in this study is compatible with the regeneration pattern of cerebrospinal fluid circulation in the organism. As long as patients can withstand, increased drainage can be more effective in removing the accumulated blood and achieving the control of the risk of complications [21]. Reference [19] also found that the LCFD method can reduce the meningeal response, achieve the control of the occurrence of cerebral vasospasm, or reduce its occurrence. This study concluded from the application that LCFD requires good perioperative nursing interventions in order to control complications. For example, it is necessary to make a detailed introduction to the patient and family members of the operation process, purpose, and function before the operation, so that the patient and family members can understand the possible risk during operation. Besides, it is necessary to prepare the required medicines such as mannitol and sedatives before the operation. During the operation, attention should be paid to the monitoring of physical signs. When the patient is found to have brain herniation, the treatment should be immediately stopped and the corresponding treatment should be carried out. In addition, the drainage operation should be performed gently and the speed of cerebrospinal fluid release should be reasonably controlled to prevent cerebral herniation [20]. After the operation, drug needs to be changed regularly, while the three-way valve should be disinfected regularly and covered with sterile gauze. In addition, the drainage bottle should be elevated before extraction, and the drainage tube should be removed only after the patient has no abnormal manifestations, and silk sutures need to be performed at the puncture site after extraction to prevent cerebrospinal fluid leakage [22].

In conclusion, continuous drainage of the lumbar cistern after intracranial aneurysm clipping can control symptoms more rapidly, reduce neurological deficits, and improve prognosis than lumbar puncture, and the drainage is safer and more widely used. However, this paper is a retrospective study, and the small number of subjects included in the study affects the representativeness and scientific validity of the results. In the future, a prospective study with a large sample and a long follow-up period is needed to fully demonstrate the difference in the effect of the two drainage methods.

## Figures and Tables

**Figure 1:** Comparison of the longest diameter of aneurysm. Compared with the longest diameter of the aneurysm in the control group, there is little difference in the observation group (*P* > 0.05).

**Figure 2:** Comparison of normalization of intracranial pressure and relief of headache. Compared with the time to normalization of intracranial pressure and headache relief in the control group, the time to normalization of intracranial pressure and headache relief in the observation group was shorter (*P* < 0.05).

**Figure 3:** Comparison of prognostic GOS evaluation. Compared with the GOS score of the control group before treatment, the observation group had little difference (*P* > 0.05) (a). Compared with the control group's GOS score after treatment, the GOS score of the observation group was lower (*P* < 0.05) (b). Compared with the GOS score before treatment in the groups, the GOS scores of the two groups were lower after treatment (*P* < 0.05) (c). *∗* indicates that the comparison is *P* < 0.05.

**Figure 4:** Comparison of cerebral artery flow velocity. Compared with the cerebral artery flow rate before treatment in the control group, there was little difference in the observation group (*P* > 0.05) (a). Compared with the cerebral artery flow rate after treatment in the control group, the cerebral artery flow rate after treatment in the observation group was lower (*P* < 0.05) (b). Compared with the cerebral artery flow rate before treatment in the groups, the cerebral artery flow rate after treatment in the two groups was lower (*P* < 0.05) (c). *∗* indicates that the comparison is *P* < 0.05.

**Figure 5:** Comparison of neurological deficit scores. Compared with the scores of neurological deficits before treatment in the control group, there was little difference in the observation group (*P* > 0.05) (a). Compared with the score of neurological deficit after treatment in the control group, the score of neurological deficit after treatment in the observation group was lower (*P* < 0.05) (b). Compared with the scores of neurological deficits before treatment in the groups, the scores of neurological deficits after treatment in the two groups were lower (*P* < 0.05) (c). *∗* indicates that the comparison is *P* < 0.05.

**Table 1:** Comparison of general information of 2 groups ($\bar{x}$ ± *s*)/[*n* (%)].

Information		Lumbar cistern group (*n* = 38)	Lumbar spine group (*n* = 37)	*t*/*X*^2^	*P*
Gender	Male	20 (52.63)	21 (56.76)	0.129	0.720
	Female	18 (47.37)	16 (43.24)		

Age (year)		60.13 ± 10.75	61.29 ± 11.12	0.459	0.647
Interval between operations (days)		1.75 ± 1.02	1.81 ± 1.06	0.250	0.803
Longest diameter of aneurysm (cm)		1.52 ± 0.49	1.55 ± 0.51	0.260	0.796
Hunt–Hess classification	Grade I	17 (44.74)	15 (40.54)	0.846	0.193
	Grade II	11 (28.95)	10 (27.03)		
	Grade III	10 (26.32)	12 (32.43)		

Aneurysm site	Internal carotid artery	10 (26.32)	11 (29.73)	0.516	0.418
	Anterior communicating artery	8 (21.05)	10 (27.03)		
	Anterior middle posterior cerebral artery	12 (31.58)	10 (27.03)		
	Vertebrobasilar artery	5 (13.16)	4 (10.81)		
	Cerebellar artery	3 (7.89)	2 (5.41)		

**Table 2:** Comparison of the total effective rate after drainage treatment between the two groups [*n* (%)].

Grouping	Cured	Got better	Invalid	Total effective rate
Lumbar cistern group (*n* = 38)	10 (26.32)	19 (50.00)	9 (23.68)	29 (76.32)
Lumbar spine group (*n* = 37)	5 (13.51)	15 (40.54)	17 (45.95)	20 (54.05)
*X* ^2^				4.102
*P*				0.043

**Table 3:** Comparison of the incidence of complications during drainage treatment between the two groups [*n* (%)].

Grouping	Hydrocephalus	Cerebral vasospasm	Cerebral infarction	Rebleeding	Other	Total incidence
Lumbar cistern group (*n* = 38)	1 (2.63)	2 (5.26)	1 (2.63)	1 (2.63)	2 (5.26)	7 (18.42)
Lumbar spine group (*n* = 37)	2 (5.41)	4 (10.81)	3 (8.11)	2 (5.41)	4 (10.81)	15 (40.54)
*X* ^2^						4.425
*P*						0.035

## Data Availability

The data used to support the findings of this study are included within the article.
